RETRACTED

# Self-Adaptation Resource Allocation for Continuous Offloading Tasks in Pervasive Computing

**DOI:** 10.1155/2022/8040487

**Published:** 2022-06-28

**Authors:** Aiman Ehsan, Khurram Zeeshan Haider, Shahla Faisal, Faisal Maqbool Zahid, Isaac Mwangi Wangari

**Affiliations:** ^1^Department of Software Engineering, Government College University, Faisalabad, Pakistan; ^2^Center of Data Science, Government College University, Faisalabad, Pakistan; ^3^Department of Statistics, Government College University, Faisalabad, Pakistan; ^4^Department of Mathematics and Computer Science, Bomet University College, Bomet, Kenya

## Abstract

Advancement in technology has led to an increase in data. Consequently, techniques such as deep learning and artificial intelligence which are used in deciphering data are increasingly becoming popular. Further, advancement in technology does increase user expectations on devices, including consumer interfaces such as mobile apps, virtual environments, or popular software systems. As a result, power from the battery is consumed fast as it is used in providing high definition display as well as in charging the sensors of the devices. Low latency requires more power consumption in certain conditions. Cloud computing improves the computational difficulties of smart devices with offloading. By optimizing the device's parameters to make it easier to find optimal decisions for offloading tasks, using a metaheuristic algorithm to transfer the data or offload the task, cloud computing makes it easier. In cloud servers, we offload the tasks and limit their resources by simulating them in a virtual environment. Then we check resource parameters and compare them using metaheuristic algorithms. When comparing the default algorithm FCFS to ACO or PSO, we find that PSO has less battery or makespan time compared to FCFS or ACO. The energy consumption of devices is reduced if their resources are offloaded, so we compare the results of metaheuristic algorithms to find less battery usage or makespan time, resulting in the PSO increasing battery life or making the system more efficient.

## 1. Introduction

Fast technology increases data and further increases user expectations on devices, including consumer interfaces such as mobile apps, virtual environments, or popular software systems. The power of the battery, therefore, charges to the advanced display, sensor, or screens that quickly consume the battery [1, 2]. The processor or devices generate large amounts of data, resulting in long delays or excessive power consumption. After all, a low latency requires increased power consumption in certain conditions. To improve the computational difficulties of smart devices with offloading, cloud computing is considered to play a significant role [3–5]. By optimizing the device's parameters so that it becomes easier to find optimal decisions for offloading tasks, a metaheuristic algorithm is used to migrate the data or to offload the task [6]. When comparing the default algorithm FCFS to ACO or PSO, we find that PSO has a lower battery or makespan time than FCFS or ACO [7]. The energy consumption of devices is reduced if their resources are offloaded, so we compare the results of the algorithms to find less battery usage or makespan time, resulting in the PSO increasing battery life or making the system more efficient [8].

RETRACTED

We have to utilize the resources or offload the task to consume time, energy cost, power consumption, and computational power, to minimize the energy usage of the smart devices we offload tasks in the cloud network and check resource parameters by using some methods [3, 9–11]. Our future job, according to the computational findings, is to offload the task using some metaheuristic algorithm combo, and the imitations conclude that the current task offloading method achieved a well-traded-off presentation between power usage ability and task execution. By applying a combo of metaheuristic algorithms using a simulator, we can check the parameters of the power usage or the job completion time [4]. To achieve energy or power consumption goals, we use cloud computing to offload the job or spread its resources. For efficiency measurements, we use metaheuristic algorithms [12, 13].

The goal of this paper is to optimize the resources for computational tasks and offload the task to the cloud server through a virtual environment. In particular, we use metaheuristic algorithms for measuring the battery time or makespan and then compare the results to investigate which strategy reduces the makespan time or uses more energy. Our main contribution is that we decreased the energy consumption/battery usage and saved the execution time of the tasks by optimally offloading them on the other resources available. For this purpose, we proposed an efficient fitness function in the metaheuristic algorithms, i.e., ACO and PSO, which guaranteed an extensive increase in the efficiency of the cloud network in lesser iterations as compared to the work done in the literature. Metaheuristic algorithms were also chosen in an optimal fashion using CloudSim to resolve energy consumption. It was done by comparing algorithms in a rigorously precise manner which yielded promising numerical results in the simulation to reduce energy, battery usage, and resource allocation. To achieve energy or power consumption goals, we have used a cloud computing advantage to offload the task as well as allocate its resources. We set the resource limit to allow for certain big computational tasks that can be performed using cloud or edge computing. The use of a metaheuristic algorithm for task offloading and the simulated results reveal the strategy of reducing the makespan time as well as energy usage at the most.

RETRACTED

## 2. Related Work

In the digital world, task offloading from smart devices to cloud servers has been considered to be a successful technique for increasing smartphone functionality and battery life [14]. Power costs and energy usage, both of which are big issues, have been used to determine the effectiveness of task offloading. These two characteristics allow smartphone devices to make informed decisions about whether or not to execute task offloading [1, 2, 15–18]. Traditional Online Code Offloading, as well as Adaptive Partitioning and Dynamic Selective Offloading, is less efficient than the metaheuristic algorithm task offloading framework [19, 20]. In this paper, we point out that, the offloading task can also be used to model one of the D2D interactions. In many research fields such as sensor communications, IoT, and device (M2M) systems, offloading can be utilized as a modern communication tool [21, 22]. Pervasive computing enables consumers to connect to an app quickly and reliably (MCC) using stratified computers. Although it is difficult to deliver complex services on low-power devices such as smartphones and tablet computers, it is possible. To resolve the problem, numerous approaches have been proposed, including implementation or structure modifications (for details, please see Table 1). They assume that just by actively splitting the request and offloading most of the execution time to either an efficient nearby proxy, this issue can be solved [12, 20, 23, 24].

### 2.1. Offloading

An automated task offloading engine cannot make its choice correctly by ignoring the operating conditions and network environment. Cloud servers used multiple methods to offload the task using servers that are the most basic or general among the computations fields [24, 25]. For the storage volume and computation size, the cloud is the most appropriate or efficient, and the latency can restrict its operation and provide the computational goal from resource-restricted to high-resource technology; a technique used to send edge servers to the cloud will improve the efficiency of the requests. It is too difficult to pick the cloud platform for the offloading algorithm [25, 26]. Single servers or several servers are used to offload the task. The advantages of offloading are shown in Figure 1. The system is the design to offload the task in a server through a wireless network for offloading [4, 23, 27–29].

RETRACTED

### 2.2. Edge with Cloud

Edge is a server for tiny device datacenters that are used. The computational power for an edge cloud is distributed by the edge servers [11, 25]. Edge computing improves the network, where the data hubs are another form of storage, for the location of the access point. The edge server is often used for the smart devices' offloading endpoint to decrease the users' power or expense. The edge computing architecture illustrates the connection between the beneficial elements of the mobile cloud computing [4, 9, 25].

### 2.3. Computational Offloading

Current findings of computational offloading typically operate on smart technologies. Energy usage or power cost is the top point of interest over the issues with the short battery time of the larger smart devices [12, 30]. The highest priority is the processing time for optimization using smart devices. We use technology for offloading the task from smart devices for available resources to consume energy or resources [31, 32]. Essentially, the offloading approach allows the developers to manually describe the intent needed for further system success. Increasing the delay or contact with static code analysis and dynamic code analysis, which makes the performance good, we use improved adaptively [4, 20]. We used some techniques such as ThinkAir or cloudlet to improve performance, which manages the virtual machine (VM) with the cloud that offloads the task of improving scalability and variance similarly [5]. A perfect environment for allocating, synchronizing, or completing the code in shifting phases may be sorted by a virtual computer or handheld cloud computing. There are two approaches to complete or comparatively code the program on the server to offload based on the customer's requirement [25]. The fine-grained approach has two methods, the coarse-grained and fine-grained.

### 2.4. Performance Metrics

The algorithms are compared on the basis of the following performance metrics.

#### 2.4.1. Makespan

It is the completion time of the last job to leave the system. Let *p*(*i*, *j*) be the execution time of the offloading task on *i*th VM of *j*th cloudlet task, and the processing time of the offloading task for *i*th VM is characterized as *l*(*i*) = ∑*p*(*i*, *j*). The independent planning job is measured as *L*_max_ = max(*L*_*I*_). This is the cloudlet VM's component. *n* > *m* means some task greater than the makespan, so we have to reduce the time of makespan. We use multiobjective optimization for makespan output that requires maximization or minimization or helps VM makespan. The number of tasks associated with *N* that offloads the number of tasks on VM such as several tasks on makespan M cloudlets and the problem of makespan minimization is considered as hard. The maximum level for feature optimization is defined in the formula. Offloading makespan is defined as *G*, where makespan time is measured with the maximum limit in the equation where the task's processing time takes the maximum limit to offload the task on VM to the cloudlet. So the link between measured makespan limit tasks and offloading is valid for all makespan offloading tasks; the optimal makespan identified with *O* is formulated by changing the relationship with task offloading based on the optimal makespan [36]. Here is the equation of makespan.

(1) $$\begin{array}{c} m\times L_{\max},\\ m\times L_{\max}>\text{G},\\ m\times O>G, \end{array}$$

where the number of task = makespan is *m*, *L*_max_ is the maximum limit = offloading of task, and*O* is the optimum.

RETRACTED

The execution time offloading task (*t* ∈ *Tt* ∈ *T*) is a term used to describe the time it takes to receive input data that is expressed (*T*_*w*_), and if *t* is the processing time, the *T*_*w*_ is defined by

(2) $$\begin{array}{c} T_{w}=\frac{\max_{i}\left(t\right)}{\underset{B}{⟶}}, \end{array}$$

where max_*i*_(*t*) shows the largest data that was received for time *t* and $\underset{B}{⟶}$ is the mean bandwidth of cloudlet VMs. The time duration of the offloading task is the sum of (*T*_*w*_ + *T*_*e*_*T*_*w*_ + *T*_*e*_).

The completion time of cloudlet virtual machine is defined by

(3) $$\begin{array}{c} T_{t}=\underset{t\in T}{\sum }\left[T_{w}+T_{e}\;\right], \end{array}$$

assumed *VM*_*i*_, *i* = 1 ⋯ *m* with the overall obtainability of cloudlet on VM denoted by *m*.

(4) $$\begin{array}{c} T_{e}=\frac{MI\left(t\right)}{MIPS\left(VM\left(i\right)\right)}, \end{array}$$

then the quantity of the success period of the offloading task. The extreme achievement period is termed the makespan, which is given as *makespan* = max(*T*_*t*−1*t*_, *T*_*t*−2*t*_, *T*_*t*−*mt*_) for a cloudlet VM task offloading [10].

#### 2.4.2. Battery Consumption

Task offloading also reduce the battery time by using an algorithm to offload the task on the cloud. Performance metrics improve the battery power. We assign the resources of the task with these performance metrics. Task offloading also reduce the battery time by using an algorithm to offload the task on the cloud. We decrease the task resources with makespan or execution time using a cloud network. To decrease makespan, or execution time, we allocate task resources to task requests. Consider *EC*_*jk*_ is the energy that the task operating on the VM absorbs. *EC*_*r*_ denotes the VM's power-consuming amount or *T*_*e*_ execution completion time [17]. The consumption of energy (EC) is measured as

(5) $$\begin{array}{c} {EC}_{jk=}{EC}_{r}.T_{e}, \end{array}$$

The total energy consumed is computed as

(6) $$\begin{array}{c} f_{2}\left(x\right)=\overset{j}{\underset{i=1}{\sum }}\overset{k}{\underset{n=1}{\sum }}{EC}_{jk}, \end{array}$$

where *j* represents the numeral jobs used and *k* represents the number of VMs used, and *f*_2_(*x*) represents the total energy used in offloading tasks by using several tasks and virtual machines.

RETRACTED

## 3. Methodology

Our motive is to reduce the resources of the devices by using the best algorithm that takes fewer resources to allocate the task. There are two approaches for allocating resources: task offloading or task scheduling using performance metrics [18]. Task offloading is the best method to offload the resources or to attain the performance metrics using the task offloading technique. We use cloud computing to provide the services of offloading the task resources with makespan, energy usage, or battery time reduction. To offload the task resources by makespan or battery processing time, we use two efficiency metrics in the cloud network. In comparison to such algorithms, cloud computing platforms use CloudSim to consume energy [24, 37]. First, we simulate the task offloading using the OMNet simulator where the task is offloading on different devices using a wireless network with cloud servers. A basic simulation is done to offload the task using the wireless network from devices to the cloud server, but we cannot distribute the resources here because there is no broker class, so later we have done our simulation in the cloud network for offloading the task resources [17, 21]. Task management in cloud computing is a core challenge that limits the system's performance. The Network CloudSim Switch, Network Datacenter, and Network Datacenter Broker include three key objects [38]. We create a datacenter in clouds, we generate a host in the datacenter, or VM is generated in the host. VMs are the virtual machines representing the cloud's smart devices. Through the cloudlets, it requests to offload the task requests [37]. If a VM cannot attain, so it sends it to another VM to accomplish the task request; we have to model tasks on a VM. We aim to evaluate the device resources with various algorithms. If a VM or device does not handle the task request, then the task transfers to another VM, so the device requires less energy and resources.

To reduce the task resources, we compare some of the algorithms for high computation. But to reduce the resources of the task for makespan or battery use, the result of the ant colony optimization algorithm or the First Come First Serve algorithm is not enough. So, we searched for the best algorithm where we get the least resource time so that we compare the outcome of these three ant colony optimization (ACO) algorithm, First Come First Serve (FCFS) algorithm, or particle swarm optimization (PSO) algorithm to allocate task resources by offloading tasks. The algorithms were implemented according to the following procedural flow whose detail is presented in Figure 2.

RETRACTED

### 3.1. Implementation through Cladism Network

Here is the first step explaining the function of setting up VM. It is the first step in launching cloudlets and virtual machines. With features such as VM ID, CPU capacity, and memory, Per VM was added. Similarly, cloudlets with a name, volume, and file size are created. Using some technique, we offload the task and utilize its resources in the simulator. In the simulation, we will be using VM, cloudlets, and cloud servers [37].

### 3.2. Using Algorithms

We will use the first come first serve algorithm as default and check its parameters after this by using ant colony optimization to minimize the makespan or battery time that will result in less time, and then we compare particle swarm optimization to decrease the battery time than ACO or resulting less time. Assign the cloudlets according to their specifications to the virtual computers, such as capacity needs and bandwidth [26].

### 3.3. Assign the Task to Cloudlets

Begin simulating the implementation of cloudlets. We can use CloudSim to simulate the task offloading, where a datacenter is created to offload the task; VM is created as a user computer hosting the required user's device to offload, where the task request is submitted to the datacenter as the cloudlets. We establish a datacenter to simulate whereby host VM is generated or cloudlets are asked to unload the task to the cloud. Cloudlets are the task requesting the request to the queue to offload the request, and the user's computer is a VM that transfers the task to offload the task resource, and the datacenter is generated to offload the task, using the datacenter as cloud storage [37, 38].

### 3.4. Selection of Algorithm Parameters

Simulating the job is a resource and now evaluating its parameters such as makespan time and battery time. These parameters are determined by positioning the VM algorithm in the simulation, sending the cloudlets to order the activity to be unloaded in the cloud, and checking its resource allocation parameters. We offload the assignment for allocating the resource in this analysis, so we use metrics of makespan to decrease the makespan period or decrease the battery power time, which increases the device's capability. According to objective characteristics, parameters such as makespan, response time, waiting time, and load are calculated or power [36].

RETRACTED

### 3.5. Analysis

Through analyzing the parameters of different cloudlets, the effect is evaluated. Using the parameters, we analyze the time of makespan or battery time. To evaluate the time that decreases the battery capacity, we can verify the makespan time. We will determine the makespan period after having the outcome of these and will also measure the battery time with less energy.

### 3.6. Task Offloading Workflow

We assign the task to request using battery usage or makespan performance metrics. It is easier to reserve the funds for allocating mission offloading. The latency requirement, energy and time required for mobile execution, the time required for cloud implementation, the input data size for cloud implementation, and the corresponding data size resulting from cloud implementation are all considered in the task offloading model. Know that there are two tasks on the computer that are the same. The work release is then said to have interruptions because cloud execution requires more energy than mobile execution and has a lower latency requirement when job offloading with cloud execution. Depending on the channel and local conditions, the amount of energy required for cloud execution varies. These considerations, however, have little impact on smartphone deployment. So, it is believed that the consumption of energy during mobile execution is steady. Either on cloud computers or a cloud server, cloud execution takes place. The energy required for cloud server execution during uplink and downlink transmission is determined by energy consumption. Based on the completion of specified data rate parameters on both input and output transfers, the latency state is fulfilled by telephone or cloud execution. It might appear like there is a single entry point for each cloudlet, and the system uses one cloudlet to offload work. However, the cloud execution process is limited in computational capacity. During the task offloading procedure, if the smartphone is outside the range of access points, the cloudlet is executed. The given data is transferred through the task offloading using cloudlet, and the output data is composed. The energy used by both the uplink and downlink during cloud execution at cloudlets is included in the total energy used during the transfers.

## 4. System Design of Offloading

In the task offloading framework with a multiobjective feature, the current task offloading architecture uses a specific optimization technique for task offloading. The new method works with competing priorities like processing time and electricity prices. The workflow in the cloud computing task offloading environment is then planned using a multiobjective task offloading model shown in Figure 3.

RETRACTED

### 4.1. Simulation Design for Offloading

Makespan and energy costs are said to maximize brand awareness by optimizing resource usage based on the minimization feature. Makespan is processed completion time and is characterized also as a combination of time consumed or process average amount in the flow. On a VM, the makespan is controlled by the task's size and computation capability, and it may be expressed using this equation: *T* = size of task/capability for computing. Energy costs were calculated as the product of the time of execution as well as the VM access rates, where it is assumed that certain every minute, cloud infrastructure is charging. *P* = VM × process time. The workflow was identified to use a series of the assigned task, and it is known as a workflow during its interconnectivity. The task offloading time needs the maximization or minimization of the resource through makespan.

### 4.2. Metaheuristic Algorithm

Metaheuristics, on either side, represent methods that are independent of an issue. As such, they will not benefit from the current problems' complexity. It is not greedy in particular. In particular, a slight regression of a method can also be tolerated the designed to simulate methodology which helps to investigate an optimal solution very systematically and therefore to achieve a better solution that can often correspond with either the best solution [6, 39, 40]. Metaheuristic would be a problem-independent method, but to apply the methodology to the nature of the problem, it will be essential to do great of all its intrinsic parameters.

In this research, we use a metaheuristic algorithm to improve the ability with the combination of hybrid algorithms.

- Nature-inspired or problem independent
- Close to the optimal solution

### 4.3. First Come First Serve (FCFS) Algorithm

First Come First Serve is an algorithm that performs queued requests and procedures immediately to arrive. That is the shortest and fastest algorithm. This algorithm is a method that allows the task to be offloaded. Energy is expended or the mission is discharged. FCFS (First Come First Serve) efficiency and enhanced FCFS discharge algorithms for complex real-time computer systems in which tasks arrive as a random process and each task have a laxity that determines the maximum time a task can wait for the operation. The key objective is to accomplish the mission of offloading to enhance the efficacy of the makespan of First Come First Serve, where makespan S1 is taken into account so that the makespan S2 for the proposed ant colony optimization enhances it and the particle swarm optimization algorithm improves the efficiency of S2 that makespan is less than the makespan of both for offloading's resulting in the offloading.

RETRACTED

### 4.4. Ant Colony Optimization

ACO was the first algorithm based on swarm intelligence. In essence, ACO mimics social ants' harvesting activity in a colony, and pheromone is used to model ants' local encounters and communications. Every ant deposits pheromones, and they eventually evaporate over time. Ant colony optimization is an optimal solution for computational problems; they find the shortest path for the food. Ants release the pheromone which is easy to find the best path [41].

- Based on swarm intelligence
- Optimal for local search

The equation of the ant colony optimization is

(7) $$\begin{array}{c} m_{ij}=\frac{{\left(T_{ij}\right)}^{2}{\left(n_{ij}\right)}^{x}}{\Sigma {\left(T_{ij}\right)}^{x}{\left(n_{ij}\right)}^{v}} \end{array}$$

where *m*_*ij*_ relates to the pheromone value to task *t*_*i*_ and resource*r*_*j*_. *n*_*ij*_ denotes the heuristic function. *x* determine the influence of pheromone value. *v* determines the influence of heuristic function. *x* is the inspired value for the pheromone, and *v* is the expected inspired value that shows the importance of heuristic function.

The algorithm of ACO is as follows:

### 4.5. Particle Swarm Optimization

The particle swarm optimization (PSO) algorithm was suggested once it was improved from several perspectives. PSO can be made more efficient by refining its iterative mechanism or by combining the initial parameters and heuristic methods with the original PSO algorithm [42]. It swarms the particle, optimizes iteratively, and tries to improve the particle position [42]. It schedules tasks on virtual machines with the goal of task scheduling tasks on virtual machines and reducing task response time [7, 43].

- Optimal for global search
- Update position or velocity
- Shortest path in a graph
- Less numb of iterations
- Fast evaluation
- Easy mathematical formulation
- Degree of imbalance close to 1

Equation of particle swarm optimization

*i* ^*th*^ where *t* is the iterations.

(*t* + 1)*i*^*th*^ Particle updates position and velocity

(8) $$\begin{array}{c} \overset{⟶}{X_{t}}\left(\text{t}+1\right)=\overset{⟶}{X_{t}}\left(\text{t}\right)+\overset{⟶}{V_{1}}\left(\text{t}+1\right). \end{array}$$

Velocity updates particles

(9) $$\begin{array}{c} \overset{⟶}{V_{1}}\left(\text{t}+1\right)=\omega *\overset{⟶}{V_{1}}\left(\text{t}\right)+C_{1}r_{1}\left(\overset{⟶}{X_{1}}-\overset{⟶}{X_{1}}\left(t\right)\right)+\left.C_{2}r_{2}\overset{⟶}{Z_{1}}-\overset{⟶}{X_{1}}\left(t\right)\right) \end{array}$$

The algorithm code for offloading using PSO is as follows [43].

RETRACTED

## 5. Results and Discussion

In CloudSim 3.03 and the NetBeans IDE, FCFS, ACO, and PSO algorithms are introduced. By taking “makespan” as a core concern, a performance function is added, and the performance index of each algorithm is measured. A broker class datacenter is used which transmits the cloudlets with the fitness value to the available virtual machine. For various tasks and virtual machines, the start time, completion time, and execution time of cloudlets are noted. CloudSim entities carry out the simulation, and their configuration is described as follows.

### 5.1. Experimental Setup and Parameter Settings

Parameters of the simulation configuration for the experimentation and the cloudlets that were used are represented in Table 2.

### 5.2. Simulation Results

In the simulator, the architecture of our simulation is built where tasks are offloaded to a separate VM ID in the datacenter. In the omnetpp simulator, where a cloud server is used as a datacenter, VM is created for hosting devices, or the wireless network that is created for accessing the VM or datacenter, and the task requests that submit the task download request are cloudlets.

For the omnetpp simulations, a system is developed that will unload the operation of computers and will increase the computing ability of machines with high capacity. We design a framework where a data server is used to offload the service; we use the cloud server as a datacenter; the virtual machine of the VM is generated for the computer of the appropriate user by a wireless network that sends tasks (see Figure 4). Cloudlets operate with the job order, and VM requests to unload the task in the datacenter to improve efficiency.

We took 200 cloudlets in the end, which are submitted on VM. The cloudlet, VM, host, and datacenter settings are kept the same. FCFS, ACO, or PSO are compared for energy consumption. This comparison table shows the time gap in makespan or battery capacity. We used metaheuristic-based algorithms to offload the task using cloudlets (0-200). ACO parameters are settled as *α* = 2, *β* = 3, *t*_*j*_ = 200, *R*_*j*_= 5 (VM), or max iteration = 100, and PSO parameters are set as *c*_1_ = 2, *c*_2_ = 2, and *w* (initial weight); it linearly varies among 0.9 to 0.03 encoding schema = matrix representation.

### 5.3. FCFS Result

The output of the 200 cloudlets is presented in Table 3 which assigns the task request to the VM that is offloading the task into the datacenter. The required files show the time before the execution or after the execution and also the start time or finish time, so the makespan time shows the less time. Here is the output of the FCFS algorithm with 200 cloudlets.

RETRACTED

The FCFS shows the battery life that comes in the order. FCFS resulting makespan time is 37.59, whereas the battery time after execution is 76.93%.

### 5.4. ACO Result

The ant colony optimization algorithm is based on the behaviors of ants seeking a passage between their colony and a food supply, and it looks for an optimum route in a network. The performance of the 200 cloudlets that assign the work request to the VM that offloads the task to the datacenter is investigated, and the results are presented in Table 4. We delegate VM IDs as a user device in the simulation to order the datacenter to unload the task by cloudlets that request the task to be unloaded in the cloud. The appropriate files often show the start time or completion time before the execution or after the execution so that the makespan time displays less time.

Here is the result generated with 200 cloudlets. ACO provides better results than FCFS; it reduced the makespan time to 30.82 or battery time to 66.77%. We attached the link to 200 cloudlets.

### 5.5. PSO Result

Now we investigate the performance of 200 cloudlets using 5 VM assigning the assignment to the datacenter so that we use the algorithm of particle swarm optimization which is metaheuristic algorithm. It is created on a shared set of N swarm-sized entities, called a swarm. We take cloudlet IDs which is assigned the request to the virtual machine; the virtual machine assigns the job to be discharged into the datacenter. We allocate VM IDs as a user computer to request in the simulation and the datacenter to unload the task through cloudlets that request the task to be unloaded in the cloud. The performance results in Table 5 indicates the time before or after the execution of the makespan time or battery use time, and the optimization algorithm for particle swarm is better for reducing the makespan time or reducing energy consumption.

PSO performance is better than ACO; it reduces makespan time by 21.78 or battery time by 44.42% (see Table 6); thus, PSO algorithm is better for increasing the efficiency of the device for computational tasks. By using PSO, it reduces the time of execution and makespan. The performance of the particle swarm optimization algorithm is found to be better than these algorithms; it reduces battery usage or enhances the ability of the device; ACO reduces the time of makespan as well as battery time, but particle swarm optimization results in improving the device.

RETRACTED

Here, initially, we took battery percentage = 99%, and then each algorithm consumed battery (battery before execution- battery after execution), e.g., in PSO (99 − 54.58 = 44.42), i.e., least in the segment, and shows PSO dominated the results of FCFS and ACO.

Finding reduced time with calculating the PSO to FCFS or PSO to ACO. Overall analysis showed that the evaluation of the time is calculated where PSO is executed time calculated by the FCFS time, so here is the formula we used to calculate the final execution time. Decrease = Original number–new number. Find makespan time and battery usage time result, so we calculate where PSO final execution time is calculated with FCFS time or ACO. PSO execution time is less than these algorithms; thus, PSO reduces more time.

Makespan time

PSO = 21.78 to FCFS = 37.59 is = 42.06%.

PSO = 21.78 to ACO = 30.82 is = 29.33%.

Battery usage time

PSO = 44.42 to FCFS = 76.93 is = 42.26%.

PSO = 44.42 to ACO = 66.77 is = 33.47%.

Our main purpose is to reduce energy consumption to increase device efficiency. Using metaheuristic algorithms, offload the task and utilize its resources for enhancing the device's capability. Particle swarm optimization reduces the time of execution more than FCFS or ACO or makes the device efficient to handle the task load. Task offloading is better to offload the tasks on the server and make the device more convenient to execute the tasks. Through metaheuristic algorithms comparison, we calculate the execution time of battery usage or makespan time so we find out the PSO is reducing more time than others.

The results in Figure 5 showing makespan time between FCFS, ACO, and PSO confirm the difference between these cloudlets, whereas the graph of battery time usage shows the reduction of battery life between FCFS, ACO, and PSO offloading which is showing the battery life using 50-200 cloudlets.

## 6. Conclusion and Recommendations

We analyze the performance of the FCFS, ACO, or PSO and find that the ACO performs better than FCFS as well as the PSO. Furthermore, the simulation results showed that the PSO reduces more energy than either of the others. The results of simulations also revealed that the time of execution power is reduced by offloading and the accuracy of job offloading is improved. The ACO makespan is 7% or energy 9.80% less than FCFS, whereas the PSO performs 9% in makespan and 22% in battery time well from ACO.

In our research, we maximize the resource utilization of the machine using heuristic algorithms that reduce the resource availability time that improve the efficiency of the machine. Such measurements help in determining the time complexity and indeed the cloud server during the offloading of the task. In the long term, it is possible to improve the proposed method by taking into consideration the probability of outages associated with real-time network metrics. Offloading is very necessary for effective usage in the cloud world. Different cloud environment offloading algorithms based on this paper are compared with algorithms and evaluated distinguishable offloading parameters such as resource allocation makespan or battery time. In some iterations, PSO and ACO fall into local optima when child tasks exist for better conversion rate and QoS awareness which is a limitation of this research. This can be further enhanced to attain a better response for global optimization in the future. The proposed work can also be implemented in the future as a hybrid of ACO or PSO, or metaheuristic methods, like cost parameters, like cost estimation, or resource usage in the cloud computing environment.

RETRACTED

## Figures and Tables

**Figure 1:** Offloading advantages.

**Figure 2:** Systematic flow adopted for offloading task.

**Figure 3:** Workflow in the cloud computing task offloading.

**Figure 4:** Offloading simulation using OMNet++ IDE.

**Figure 5:** Graphical representation of makespan and battery time.

**Algorithm 1:** Ant Colony Optimization (ACO).

**Algorithm 2:** Particle Swarm Optimization PSO.

**Table 1:** Evaluation table.

Author Year	Method	Purpose	Description
Erana Veerappa Dinesh Subramaniam	Gray wolf optimization	In the current time, task offloading from smartphones to cloud servers has proven to be a promising technique for increasing smartphone functionality and battery life. The cost of communication and energy usage are used to determine the effectiveness of task offloading [17]	Strength We offer a new framework that uses a task scheduler to reduce energy usage during HMCC task offloading [10]. The suggested system uses a multiobjective function to model the scheduler, which takes into account network metrics, cloud parameters, and other system data Weakness The outcome in tangling also not accurate result in global optimization. Low precision or poor local optimization
Kaiyang Liu (2016) [18]	An iterative decoupling algorithm	Internet of things offers a new concept to improve the abilities through offloading the computational resources to consume less energy from smart phones; we offload resources to cloud server.	Strength To use less energy, the users of smart devices offload work with an appropriate data connection and contact efficiency, and offloading decision strategy is studied Weakness It takes large computation period
Kai Lin (2018) [23]	Fruit fly algorithm	An offloading algorithm fruit fly is suggested to enhance the distribution by offloading and utilizes its resources to achieve less energy usage under responsibilities assigned. Energy consumption, time, and cost efficiency, relative to cooperative multitask, allocated total on an ant colony optimization algorithm and algorithm based on the heuristic server. The findings further suggest the efficiency of the algorithm suggested by contrasting that with current algorithms	Strength The simulation outcomes show that the average FOTO algorithm promises better energy efficiency, reduced processing times, and also reduced datacenter costs which are used for edge computing in advanced applications. For further study into mobile offloading across numerous mobile devices, a cooperative device-to-device communication system will be established, allowing mobile devices to assist each other in offloading duties. This method can increase channel capacity while maintaining high bandwidth efficiency, allowing task offloading to be better utilized Weakness Less accuracy or bad optimal solution
Jing Zhang, Weiwei Xia (2018) [3]	Subalgorithms	Low power consumption and low computing capacities restrict the installation of high computational programs on smart devices	Strength The appropriate approach that impedes efficiency that analyzes the characteristics will transfer the intensive apps as on a cloud Weakness Problem not solving independently
Men his chin, Ben Liang, Min dong (2016)	Heuristic algorithm	Each smartphone user requires several independent tasks that share the resource while offloads workload to the cloud network for less computational power through other methods [33]	Strength Currently, we work on improving the offloading and allocating contact tools for all projects, to eliminate electricity expenses, computing costs, and delays for all consumers. Our approach can be applied to several users and activities where even the machine sophistication of thorough search becomes costly Weakness This method is not providing optimal solution
Rahul Yadav (2020) [34]	Heuristic approach	To solve the energy consumption and resource allocation problem in this paper used an energy efficient computation.	Strength It is better for the energy saving, latency, and energy latency cost than overall schemes [34]
Muhammad Shafiq (2021) [35]	RL based	Computation Offloading using Reinforcement Learning (CORL) For more energy, less battery time, and delay in portable machines, there are not enough resources for allocate these, so in this research, we proposed some work to handle this situation	Strength Better offloading decisions in a quick time [35]

RETRACTED

**Table 2:** Experimental setup and parameter settings.

Virtual machine parameter	Size = 10000; image size Int ram = 512; VM memory Int MIPS = 1000
Cloudlets constraints	Length = 500 File size = 300 Output size = 300 Pe′s number = 1
Number of datacenters	1
Number of VM	5
No of cloudlets	100-500
Nature of cloudlets	Independent
Performance metrics analysis	Makespan or battery usage
Hardware configuration	Processor: Intel (R) Core ™ i3 -2310 M CPU@ 2.10GHz Hard disk: 1 TB Ram: 2 GB.
Software configuration	Operating system: Windows 10pro Simulation software for offloading: omnetpp Simulation software for resource allocation: CloudSim 3.03 IDE: NetBeans: 8.1 Java version: JDK 1.8-172

**Table 3:** Yielded values for FCFS.

Cloudlet ID	Status	Priority	Datacenter ID	VM ID	Time	Start time	Finish time	Input file size	Output file size	Battery before exec	Battery after exec	Required files
0	Success	4	2	0	0.11	37.15	37.26	30000	30000	99	98.84	7.766917
1	Success	1	2	1	0.11	15.45	15.56	30000	30000	98.84	98.28	28.47368
2	Success	4	2	2	0.11	36.27	36.38	30000	30000	98.28	97.92	17.94737
98	Success	1	4	18	0.11	16.31	16.42	30000	30000	61.13	60.69	22.09774
99	Queued	3	4	19	-1	0	-1	30000	30000	60.69	60.39	14.66917
197	Queued	4	4	17	-1	0	-1	30000	30000	22.91	22.88	1.691729
198	Queued	3	4	18	-1	0	-1	30000	30000	22.88	22.19	34.65414
199	Queued	2	4	19	-1	0	-1	30000	30000	22.19	22.07	5.864662
						Makespan 37.59				Battery usage 99-22.07		76.93

**Table 4:** Yielded values for ACO.

Cloudlet ID	Status	Priority	Datacenter ID	VM ID	Time	Start time	Finish time	Input file size	Output file size	Battery before exec	Battery after exec	Required files
0	Success	1	2	0	0.11	21.46	21.57	30000	30000	99	98.92	20.55639
1	Success	4	2	1	0.11	12.15	12.26	30000	30000	98.92	98.79	28.30075
2	Queued	3	2	2	-1	0	-1	30000	30000	98.79	98.68	36.5188
	—				—				—		—	
98	Queued	2	4	18	-1	0	-1	30000	30000	68.13	67.69	26.80451
99	Queued	2	4	19	-1	0	-1	30000	30000	67.69	67.39	27.30827
100	Success	5	2	0	26.26	0.2	26.46	30000	30000	67.39	67.18	26.26316
	—				—				—		—	
197	Queued	3	4	17	-1	0	-1	30000	30000	32.96	32.82	4.210526
198	Queued	2	4	18	-1	0	-1	30000	30000	32.66	32.47	17.07519
199	Queued	4	4	19	-1	0	-1	30000	30000	32.47	32.23	17.96241
						Makespan 30.82			Battery usage 99-32.23		66.77	

**Table 5:** Yielded values for PSO.

Cloudlet ID	Status	Priority	Datacenter ID	VM ID	Time	Start time	Finish time	Input file size	Output file size	Battery before exec	Battery after exec	Required files
0	Success	4	2	0	0.11	6.42	6.53	30000	30000	99	98.94	3.165414
1	Success	4	2	1	0.11	16.24	16.35	30000	30000	98.94	98.82	28.2406
2	Success	3	2	2	0.11	9.05	9.16	30000	30000	98.71	98.59	9.458647
	—		—				—		—			
98	Success	3	4	18	0.11	11.23	11.34	30000	30000	79.11	78.88	36.90977
99	Success	5	4	19	0.11	17.55	17.66	30000	30000	78.88	78.62	22.96992
100	Success	4	2	0	0.11	6.64	6.75	30000	30000	78.62	76.28	33.73684
	—		—				—		—			
198	Queued	3	4	18	-1	0	-1	30000	30000	54.87	54.74	10.45113
199	Queued	5	4	19	-1	0	-1	30000	30000	54.74	54.58	12.85714
						Makespan 21.78				Battery usage 44.42		99-54.58

RETRACTED

**Table 6:** Results comparison calculations.

No. of cloudlets	FCFS		ACO		PSO	
	Makespan	Battery usage	Makespan	Battery usage	Makespan	Battery usage
	(in sec.)	(in %)	(in sec.)	(in %)	(in sec.)	(in %)
50	9.39	99 − 88.28 = 10.72	7.7	99 − 90.95 = 8.05	5.8	99 − 92.06 = 6.94
100	18.82	99 − 66.21 = 32.79	15.51	99 − 80.01 = 18.99	10.89	99 − 84.89 = 14.11
150	27.8	99 − 45.94 = 53.06	22.72	99 − 60.02 = 38.98	16.33	99 − 70.78 = 28.22
200	37.59	99 − 22.07 = 76.93	30.82	99 − 32.23 = 66.77	21.78	99 − 54.58 = 44.42

## Data Availability

The data can be requested from the corresponding author.
